The article "Exposure to Sex Education and Its Effects on Adolescent Sexual Behavior in Nigeria" was published in 2022. Journal: J Environ Public Health.

# Exposure to Sex Education and Its Effects on Adolescent Sexual Behavior in Nigeria

**DOI:** 10.1155/2022/3962011

**Published:** 2022-06-01

**Authors:** Uyi E. Osadolor, Emmanuel O. Amoo, Dominic E. Azuh, Ikono Mfonido-Abasi, Christian Philip Washington, Oke Ugbenu

**Affiliations:** Demography and Social Statistics, Department of Economics & Development Studies, Covenant University, Km 10, Idiroko, Ota, Nigeria

## Abstract

Sexual behavior during adolescence fundamentally steers the future life of both girls and boys, and it should be guided with appropriate education, especially as it also represents a key factor to be considered in attainment of sustainable developmental goals. The study assessed the effect of exposure to sex education on adolescents' sexual behavior. The primary and cross-sectional survey data used for this study were analyzed using basic descriptive statistics and binary logistic regression analytical technique. The results, among others, highlighted that the most common sources of first sex education among the respondents are school (54.6%), family (21.6%), social media (9.5%), and others like television (7.6%) and books or magazines (4.9%). Frequency of discussion on sexual matters is positively associated with the use of protection such as condom (*β* = 0.261; *p* ≤ 0.01). The study gave support to the increasing pursuit of sexuality education. However, since adolescents' needs could vary by demographics, streamlining sex education need by age and sex characteristics could enhance its effectiveness.

## 1. Introduction

Sexual behavior during adolescence fundamentally steers the future life of both girls and boys. It should be guided with appropriate education, especially as it also represents a key factor in the attainment of sustainable developmental goals. It is estimated that over 21 million adolescents aged 15–19 years get pregnant annually in low economies [1–3]. At the same time, over 50% of them give birth, excluding additional 777,000 adolescents that are less than 15 years who give birth in developing countries [4]. The health issues and consequent challenges associated with sexual lifestyles and behavior among adolescents are enormous. It is reported that over 3.9 million girls between the ages of 15 and 19 carry out unsafe abortions annually worldwide [5]. Other literature indicates that young people aged 10–19 represents relatively 4% among the population living with HIV infection [6].

Although Africa does not have the largest number of adolescents globally, adolescents make up the most significant proportion of the population of the sub-Saharan African region, with relatively 23% of the region's population aged 10–19 years [7]. In sub-Saharan Africa, nearly four times as many girls aged 10–19 were infected with HIV than their male counterparts in 2018 alone [7]. Specifically, adolescent sexual behaviors have been linked to a number of life events, and several health challenges, for example, early pregnancy, risks of pregnancy-related mortality, delivery complications, infant mortality, adolescent fatherhood, and school dropout [8,9]. Sex education therefore portends greater potential in preventing and reducing these risks [8,9]. Sex education could enlighten the adolescent on the avoidance of pregnancy, HIV, other sexually transmitted infections, including other chronic health conditions and disabilities that are linked to adolescent sexual behavior [8–10]. Thus, constant assessment of sexual education among adolescents cannot be overemphasized.

The article "Exposure to Sex Education and Its Effects on Adolescent Sexual Behavior in Nigeria" was published in 2022. Journal: J Environ Public Health.

Every year, approximately 20 million new cases of sexually transmitted diseases are reported with 50% of the cases occurring among adolescent aged 15–24years [11,12]. It has also been estimated that 25% of all sexually active female adolescents have experienced one or more forms of sexually transmitted infection, with the most common as human papillomavirus and *Chlamydia trachomatis*. Sexually transmitted infections have established as major cause of morbidity among women and men that has potential for high risk human papillomavirus (hrHPV) infections which in chain-like reaction could spur cervical cancer [13]. While the identification of STIs as co-factor of cervical cancer in most women that are HPV-positive (Martinelli et al. [13]) cannot be treated with levity, the evidence of similar linkage betweenSTD trichomoniasis and prostate cancer [14] should call for serious concern in public health domain. This buttresses the fact that adolescent sexual behaviour that could trigger sexually transmitted diseases should be paramount to health and wellbeing stakeholders.

The fact that the rate of sexually transmitted infections is on the increase in both adolescent males and females [11,12] sends a signal that immediate and sustained intervention would be necessary to enhance the future health of the population and economic productivity. It is highly needful that a child receives sex education considering the fact that naivety can breed unwanted outcomes [15,16]. A systematic review study to evaluate the effectiveness of sex education intervention showed that sex education had a positive effect on adolescent sexual behaviour [17].

Since the approval and introduction of sexuality education policy in Nigeria in 1999 with curriculum modification that teaches sexuality education [18], the efficacy is with mixed results. Till date, there is increasing concern on high rates of adolescent pregnancies and spread of STDs and STIs [19]. The fertility rate of 104 births per 1000 among Nigeria's adolescents' women aged 15–19 is one of the highest in the world [20]. This includes a galloping increase in STDs such as chlamydia, genital herpes, genital warts, gonorrhea, some forms of hepatitis, syphilis, and trichomoniasis with HIV as the most prominent [20]. At 2012, a study on adolescents in the secondary school has reported that 55.7% and 21.9% of boys and girls engaged in masturbation in the study location [16]. A near recent study conducted by the Resource Centre for Adolescence Pregnancy Prevention (ReCAPP) reported that about half of adolescents engage in oral sex and one out of 10 adolescents practices anal sex [21]. The recent trends have made the issues of early sexual debut worrisome in Nigeria and including other sub-Saharan African countries. Amoo [22] reported men's median age at first sex as 18 for Nigeria and Ethiopia and 16 for Zambia while adding that the median age at first marriage for women in Ghana, Kenya, and Zambia is relatively 17 [23]. Similar report by Durowade et al.[19] highlighted that the average age at first intercourse among adolescent as 15 years. In 2003, the Nigerian Association for the Promotion of Adolescent Health and Development (NAPAHD) informed the public that adolescents accounted for 80% of complications during abortion procedures [24]. Considering the conspicuous risk of sexual behaviour and their outcomes among the adolescent gives doubt to the coverage and impacts of sex education in developing nations, especially in Nigeria where adolescents constitute relatively 22% of the population and the rising wave of STIs among them.

The article "Exposure to Sex Education and Its Effects on Adolescent Sexual Behavior in Nigeria" was published in 2022. Journal: J Environ Public Health.

A study conducted in a state in Nigeria showed that less than a quarter of the respondents were exposed to sex education and over two-thirds of them have engaged in early sexual activity [19]. With respect to the various reports of the adolescent sexual behaviour in Nigeria, there seems to be inadequate, inappropriate guidance, although colossal extinction of the 1999 sexuality education policy cannot be confirmed. Lack of education on sexual behavior among the adolescents or its ineffectiveness is inimical directly or indirectly to adolescent education, future engagement in economic activity, and their wellbeing and poverty or wealth level in the country. This study, therefore, aims to assess the exposure to sex education from different media and the varying effects it could have on the sexual behavior of adolescents in Nigeria. This would be essential to quantify health effects and spur prompt interventions or decision to prioritize relevant actions.

The article "Exposure to Sex Education and Its Effects on Adolescent Sexual Behavior in Nigeria" was published in 2022. Journal: J Environ Public Health.

## 2. Materials and Methods

### 2.1. Study Design, Area, and Period

We conducted a survey-based study among adolescents aged 10 to 19 years who were in their first year across the seven faculties of the Rivers State University in Port Harcourt, Nigeria. A total of 3780 first year university students were registered with the University. Data were collected between March 1 and 31, 2021.

### 2.2. Sample Size Determination and Sampling Procedure

The theoretical sampling frame used was the 3780 number of first year students reportedly registered as obtained from the university registry. We therefore calculated the sample size adopting the sample size determination method of Taro Yamane as adopted by Adekola et al. [25]. Using a sampling error of 0.05, the computation yielded a sample size of 362. The study employed the use of simple random sampling in order to select adolescent participants (aged 10–19 years) during the study period. Lecture schedules (timetable) were followed as guide, and random selection of respondents was conducted among volunteered students in randomly selected lecture rooms.

### 2.3. Study Variables

The dependent variable is a variable of sexual indicator measured as “having sexual partner.” Sexual behavior refers to experiences and expression of sexuality and conceptualized in this study as “having sexual partner.” The independent variables were socio-demographic factors such as age, gender, religious affiliation, education attainment, usual place of residence, and parental factors (e.g., father's occupation, mother occupation, respondent's living arrangement, and parent's education). The intervening variable for this study was the exposure to sex education.

### 2.4. Data Collection Procedures

Data were collected from the sampled population through the use of a self-administered questionnaire. The study participants were educated on the objective and purpose of the study and the likely contribution of the study to the society. Daily filled questionnaires were collected and checked for consistency and completeness. To ensure data quality, data collection instruments were given high emphasis during design, and the questions were pretested. The principal investigator conducted training for data collectors on the methods of data collection. The pretesting of the questionnaires was conducted two weeks before the commencement of the main survey.

### 2.5. Data Processing and Analysis

The entire questionnaires were checked and entered into the IBM SPSS statistics for analysis. Three levels of analysis were employed, namely, a univariate, bivariate, and multivariate analyses. The univariate analysis was used to profile the socio-demographic profiles of the respondents. The bivariate analysis was used to understand the association between the selected socio-demographics variables and having sexual partner. In addition, the exposures to sex education variables were cross-tabbed with having sexual partner. Two hypotheses were formulated for this study and are presented in alternative forms; namely, (1) adolescent background characteristics significantly influence adolescent exposure to sex education, and (2) there is a significant relationship between exposure to sex education and certain sexual behavior among adolescents. Binary logistic regression employed tested the effect of the exposure to sex education on having a sexual partner, and the effect of socio-demographic characteristics on having a sexual partner. The adjusted odds ratio at a 95% confidence interval was adopted to determine the strength of association between the dependent and each of the independent variables.

The article "Exposure to Sex Education and Its Effects on Adolescent Sexual Behavior in Nigeria" was published in 2022. Journal: J Environ Public Health.

### 2.6. Ethical Consideration

Ethical clearance was obtained from Covenant University Health Research Ethics Committee (Ref: CHREC/061/2021). The official letter that explains the objectives, rationale, and expected outcomes of the study was written to the Chairman Health Research Ethics Committee, Covenant University. Prospective respondents who were under legal age (<18 years old) were introduced to the assent form while consent forms were dully approved by supervising faculty of the department or lecture coordinators. However, students whose parents could be reached were contacted through phone calls for permission. The aim of the study was explained to all participants, and assurance was given on confidentiality of their responses and anonymity in publication of the reports of this study. We omitted any personal identifier from the questionnaires and maintained confidentiality of information also in this study.

## 3. Results

### 3.1. Demographic Characteristics of Respondents

Out of the 362 randomly selected adolescents, useable questionnaire was 345 (implying a response rate of 95.3% and an attrition rate of 4.7%). Relatively, 60% of the participants, 206 (59.7%), were females. The mean age was 17.80 (±2.65) years, and the majority of them, 265 (76.8%), were in the age group of 15–19 years. Above two-thirds of them, 239 (69.3%) belonged to nuclear family structure, and 262 (75.9%) lived with both parents. Results on the selected parental information show that 42.0% and 43.8% of adolescents have fathers and mothers who had attained secondary level of education, respectively (as shown in Table 1). More than half of the mothers, 59.8%, engaged in trading/services, while 44% of their fathers were civil servants (Table 1).

The article "Exposure to Sex Education and Its Effects on Adolescent Sexual Behavior in Nigeria" was published in 2022. Journal: J Environ Public Health.

### 3.2. Adolescents' Knowledge of Sex Education and Sexual Practices

Four-fifths of the respondents had discussed or read certain things on sexual matters. However, relatively half of the respondents have discussed sexual issues with relations or parents as shown in Table 2. Most respondents reported they are not frequently discussing/reading sexual matters; 90.8% have heard or read about sex education, but only 4.6% indicated they have a good knowledge of sex education as shown in Table 2. Relatively, 54.6% indicated that they first heard or read about sex education from the school. More than half of the respondents knew about STIs (95.3%), and almost half (44.6%) have knowledge of sexual activities (Table 2). Two hundred fifty-five (80.7%) know about oral sex, 58.3% know about anal sex, and 72.4% know about masturbation. Further analysis revealed that 81.2% of adolescents are aware of contraceptive use, as shown in Table 2.

### 3.3. Adolescents' Sexual Behavior and Experience

Less than half of the respondents, 140 (41.9%), had experienced sexual intercourse. Relatively 13.8% of the respondents below the age of 14 have had sexual intercourse, while 51 (15.3%) respondents aged between 15 and 19 years have had sexual encounters. Out of all the respondents who had engaged in kissing, vaginal, and anal sex, only 105 (34.1%), 126 (60.1%), and 264 (93.3%), respectively, have never engaged in any of the above sexual practices.

Questions on where their first sex experience took place revealed that 57 (42.9%) had their first sexual experience in their partner's houses, while 96 (77.4%) of respondents had between one to two sexual partners, and condom 73 (67%) was the most used type of contraceptive. 11 (47.8%) of the respondents aged 17-18 years had been pregnant or had impregnated someone as shown in Table 3.

### 3.4. A Binary Logistic Regression Illustrating the Interrelationship between Having Sexual Partner (Dependent Variable) and Selected Demographic and Exposure to Sex Education Variables

The first hypothesis tested the interrelationship between having sexual partner (dependent variable) and selected demographic and exposure to sex education variables. Binary logistic regression was employed with a binary coded dependent variable (having sexual partner) as dependent variable. The independent variables include respondents age, gender, usual place of residence, educational attainment, father's and mother's occupation, discussion/reading on sexual matter, family type, indicators of discussion of sexual issues (parents, relations), and read sexual matters. Discussion on sexual matters at any every level as captured in the study is significantly negatively related to having sexual partner (*p* ≤ 0.05).

The article "Exposure to Sex Education and Its Effects on Adolescent Sexual Behavior in Nigeria" was published in 2022. Journal: J Environ Public Health.

Respondents aged ≤14years are 0.2800 times less likely to have a sexual partner compared to older respondents aged 15–19 (*B* = −1.23; OR = 0.28). Respondents who discuss sexual issues with parents are 3.93 times more likely to have a sexual partner than those who do not discuss with a parent. However, respondents who discuss sexual matters with a relative were less likely to have a sexual partner compared to the reference category (individual who do not discuss with a relative (*B* = −1.34; OR = 0.26). The result of the analysis on parental occupation shows that adolescents whose parent are farmers are 0.12 times less likely to have sexual partner compared to adolescent whose parents are in other types of occupation. Only farming/others with respect to mother's occupation produced a statistically significant result (*p* < 0.05). This category of respondents is also less likely to have sexual partner compared to other two occupation categories: civil servant (RC) and trading/services (*B* = −2.15; OR = 0.12). Respondent's parents highest school level is statistically insignificant to having a sexual partner (*p* > 0.05). Father's occupation is positively related to having asexual partner. Farming/others amongst fathers increased the odds of having sexual partner by 1.74 times (Table 4).

Respondents who live in an urban area are 2.71 times more likely to have a sexual partner than those living in a rural area (RC) (*B* = 0.20, *p* > 0.05). Also, respondents from nuclear families had almost half the odds of having sexual partner compared to those from extended families (RC), (*B* = −0.60; OR = 0.55; *p* > 0.05). Female respondents are more likely to have a sexual partner than male respondents (*B* = 0.09; OR = 1.09; *p* > 0.05). Those who read/discuss sexual matters are less likely to have a sexual partner than those who do not read/discuss sexual matters (Table 4).

### 3.5. Logistic Regression Analysis Illustrating the Influence of Selected Factors of Exposure to Sex Education on Having Sexual Partner(s)

The binary logistic regression analyzed the relevance and interaction between the dependent variable and selected exposure to sex education variables for hypothesis two. The dependent variable is having sexual partner, while the selected independent variables are reading/discussion on sexual matters, frequency of discussion/reading on sexual matters, ever discussed sexual matters with any or both parents, ever discussed sexual matters with any relation, conceptual understanding of sex education, and source of first sex education.

The article "Exposure to Sex Education and Its Effects on Adolescent Sexual Behavior in Nigeria" was published in 2022. Journal: J Environ Public Health.

The finding shows that the odds of discussing sexual matters are significantly related to having sexual partner. Adolescents who discuss sexual matter very often were less likely to have sexual partners than those who are not discussing sexual matters (*B* = −1.01; OR = 0.36; *p* < 0.05). Similarly, adolescents who do not discuss sexual matters very often were less likely to have a sexual partner than those who do not. Discussion of sexual issues with either parents or relatives is significantly related to having sexual partner. At the same time, those who discuss sexual issues with parents are more likely to have a sexual partner than those who do not (*B* = 1.27; OR = 3.54). Those who discuss sexual issues with a relative were less likely to have a sexual partner than those who do not discuss with a relative (*B* = −1.274; OR = 0.28).

Furthermore, the result revealed that adolescents who read/discuss sexual matters were less likely to have a sexual partner than people who do not (*B* = −1.05; OR = 0.35; *p* > 0.05). Respondents who have a good understanding of sexual concepts are less likely to have a sexual partner than those who have little understanding (*B* = −1.75; OR = 0.17).

The analyses show that adolescents who source their first sex education from the various forms of media (radio, television, and social media) are less likely to have a sexual partner than those who receive it from books/magazines (RC). Adolescents whose first source of sex education is from the family and school are more likely to have a sexual partner than those who receive it from magazines/books (Table 5).

## 4. Discussion

The study provided empirical analysis of sex education awareness and knowledge among adolescents that have sexual partner and their different sexual activities in the context of university undergraduates. The study could have significant contributions in spurring initiatives or policy towards curing high-rate unwanted pregnancy, unsafe abortion, school dropouts, and SIT, HIV including young mother's death and infant mortality [18]. The study gave support to increasing pursuit of sexuality education that could enhance healthy adolescenthood, healthy sexual decision-making, and wellbeing [26].

Specifically, the study provided insight on the exposure of adolescents to sex education from different media and the varying effects things as such could have on the sexual behavior of adolescent. The study revealed that 4 out of every 10 adolescents have experienced sexual intercourse and that male adolescents are more involved in sexual risk behavior than the female adolescents. While the finding could be in tandem with previous studies [27]; [28], it signals that (1) such finding is still relevant today, and (2) the understanding of the report could spur paradigm shifts in existing strategies or their modifications. Therefore, in as much as the focus of this study is not directly to evaluate international, national, or local strategic framework on Adolescent Reproductive Health Programs, the results herein are evidences of nonabsolute success of these programs, and a need for change is imperative. The parents or guidance could also have little or no attention to male sexual behavior [29, 30], and [31, 32].

The article "Exposure to Sex Education and Its Effects on Adolescent Sexual Behavior in Nigeria" was published in 2022. Journal: J Environ Public Health.

The result in this study with adolescents aged (10–19) showed that more than half of the adolescents interviewed had engaged in sexual activities; it does not only validate past studies, but it also signals to the present prevalence rate [33–40]. The authors saw relevance in sex education and adolescents' access to adequate information as important agenda that should be vigorously pursued by stakeholders in adolescent health. The fact that age is significantly associated with having a sexual partner could be understood as natural development. As adolescents reach puberty, they tend to want to try out new things and experience things for themselves [41–45]. The profound information about the associate linkage between STIs, HPV and potential for cervical and prostate cancers [13,14] should make sexual education and adolescent sexual behaviour a serious concern in public health domain.

Notwithstanding, the highlight that adolescent discussion with parent is negatively related to early sexual debut may not be sustained taking lesson from other studies [46–50]. This finding also could be due to sacrilegious perspective of sexual issues in sub-Saharan Africa. Sexual discussion is perceived as taboo, and, when done, it is only permissible among the adults [51]. Besides, it is general erroneous believe that exposing adolescents to sex education could introduce them to early sexual behaviors or make them promiscuous [52–54]. Notwithstanding, the study extol the virtue of sexual matter discussion among adolescents as it enhances the use of protection against STI, HIV, and other venereal diseases [41,55–59].

## 5. Conclusions

The empirical analysis from the study suggests sex education awareness and knowledge among adolescentsare indispensable in the drive towards the control and prevention of sexual transmitted diseases, unwanted pregnancy, unsafe abortion, school dropouts, and SIT, and HIV, including young mother's death and infant mortality. The study concludes that the identification of multiple sexual partnership among the adolescents and retrospective years of first intercourse and the absolute effectiveness of existing sex education policy could be controversial. Adolescents would therefore require increase in enlightenment to effect a paradigm shifts in the current observed sexual behavior if attainment of health-for-all agenda is paramount to the stakeholders. While exposure of adolescents to sex education might not prevent them from engaging in sexual activities, it could equip them with required knowledge of protection against detrimental risk sexual activities that could spur ill-sexual health. Parental discussion of sexual matters with adolescents could be of importance and should not be taken lightly as incomplete information might be misleading. It is important that adolescents receive accurate information. However, since different age groups of adolescents could have different needs, the educator will need to streamline sex education based on age differences. The study gave support to increasing pursuit of sexuality education.

The article "Exposure to Sex Education and Its Effects on Adolescent Sexual Behavior in Nigeria" was published in 2022. Journal: J Environ Public Health.

### 5.1. Limitations of the Study

The study is based on self-administered questionnaires that are characterized by economical truthfulness of the data. However, the reliability test and high level of education of the respondents being undergraduates of ivory tower educational setup enhance the participant understanding of the questions and accurate responses with minimal attrition level (4.6%).

### 5.2. Novelty of the Study

This paper is novel because it contributes to the current understanding of how exposure to sex education from different media could be used to control adolescent sexual behavior in the study location that was scantily available. The holistic analysis of this study added to the existing research by identifying key components that influence adolescent sexual behavior considering the fact that analyzing the importance of these components has not been exhaustive in the literature. This paper confirms existing literature that also emphasized the crucial role of certain media of sex education such as social media, school, and television. However, the present study also identified socio-demographic characteristics such as place of residence, family type, gender, and age as significant characteristics influencing adolescent sexual behavior [60, 61].

## Figures and Tables

**Table 1:** Demographic characteristics of respondents.

Selected variables	Frequency	Percent
Place of residence		
Urban	310	89.9
Rural	35	10.1
Total	345	100
Age group		
Below 15	80	23.2
15–19	265	76.8
Total	345	100
Father's occupation		
Farming/others	76	22.4
Trading/services	114	33.6
Civil servants	149	44
Total	339	100
Gender		
Female	206	59.7
Male	139	40.3
Total	345	100
Living arrangement		
Both parents	262	75.9
Father only	13	3.8
Mother only	38	11
Other relations	32	9.3
Total	345	100
Family type		
Nuclear	239	69.3
Extended	106	30.7
Total	345	100
Religion		
Christian	331	95.9
Islam	10	2.9
Others	4	1.2
Total	345	100
Mother's occupation		
Farming/others	37	10.8
Trading/services	205	59.8
Civil servants	101	29.4
Total	343	100
Mother education		
Primary/none	91	26.4
Secondary school	151	43.8
Higher institution	103	29.9
Total	345	100
Father education		
Primary/none	77	22.3
Secondary school	145	42
Higher institution	123	35.7
Total	345	100

Source: author's fieldwork (2021).

The article "Exposure to Sex Education and Its Effects on Adolescent Sexual Behavior in Nigeria" was published in 2022. Journal: J Environ Public Health.

**Table 2:** Adolescents' knowledge of sex education and sexual practices.

Selected variables	Frequency	Percent
Discussed sex issues with relations		
Yes	170	50.0
No	170	50.0
Total	340	100
Discussed sex issues with parent		
Yes	149	43.8
No	191	56.2
Total	340	100
Knowledge of STIs		
Yes	303	95.3
No	15	4.7
Total	318	100
Oral sex		
Yes	255	80.7
No	61	19.3
Total	316	100
Read/heard of sex education		
Yes	295	90.8
No	30	9.2
Total	325	100
Knowledge of sex education definition		
High	9	4.6
Average	62	32.0
Low	123	63.4
Total	194	100
Knows masturbation		
Yes	231	72.4
No	88	27.6
Total	319	100
Discuss or read on sex matters		
Yes	276	80.7
No	66	19.3
Total	342	100
Knowledge of contraceptive		
Yes	272	81.2
No	63	18.8
Total	335	100
Knows other sexual activities		
Yes	131	44.6
No	163	55.4
Total	294	100
Anal sex		
Yes	180	58.3
No	129	41.7
Total	309	100
Source of first sex education		
School	179	54.6
Family	71	21.6
Radio	6	1.8
Television	25	7.6
Social media	31	9.5
Magazine/book	16	4.9
Total	328	100
Frequency of discussion/reading on sex		
Very often	59	17.4
Not often	151	44.5
Rarely	78	23.0
Not at all	51	15.0
Total	339	100

Source: author's fieldwork (2021).

**Table 3:** Adolescents' sexual behavior and experience.

	Frequency	Percent
Ever experienced sexual intercourse		
Yes	140	41.9
No	194	58.1
Total	334	100
Kissing practice		
Very often	70	22.7
Often	41	13.3
Not often	92	29.9
Not at all	105	34.1
Total	308	100
Vaginal sex practice		
Very often	21	7.2
Often	36	12.3
Not often	60	20.5
Not at all	176	60.1
Total	293	100
Anal sex practice		
Very often	4	1.4
Often	5	1.8
Not often	10	3.5
Not at all	264	93.3
Total	283	100
Place of 1st intercourse		
School	14	10.5
Hotel	13	9.8
Partner's house	57	42.9
Your house	40	30.1
Others	9	6.8
Total	133	100
Age at 1st pregnancy/impregnated someone		
15-16	3	13.0
17-18	11	47.8
19-20	9	39.1
Total	23	100
Action on pregnancy		
Abort	20	83.3
Keep the pregnancy	4	16.7
Total	24	100
Current sexual partner		
1-2 partners	96	77.4
3-4 partners	10	8.1
5 partners and above	18	14.5
Total	124	100
Age at first sexual intercourse	Freq	Percent
≤14years	46	13.8
15–19	51	15.3
Did not know/never	237	71.0
Total	334	100
Oral sex practice		
Very often	15	5.2
Often	19	6.6
Not often	41	14.3
Not at all	211	73.8
Total	286	100
Masturbation practice		
Very often	9	3.2
Often	8	2.8
Not often	31	10.9
Not at all	237	83.2
Total	285	100
Other sexual practice		
Very often	2	0.8
Often	1	0.4
Not often	5	1.9
Not at all	253	96.9
Total	261	100
Lifetime sexual partners		
1-2 partners	81	59.6
3-4 partners	26	19.1
5 partners and above	29	21.3
Total	136	100
Use of contraceptive		
Yes	98	30.9
No	219	69.1
Total	317	100
Contraceptives usage		
Very often	37	12.1
Not often	44	14.4
Rarely	26	8.5
Not at all	199	65
Total	331	100
Type of contraceptive used		
Condoms	73	67
Pills	33	30.3
Others	3	2.8
Total	109	100

Source: author's fieldwork (2021).

The article "Exposure to Sex Education and Its Effects on Adolescent Sexual Behavior in Nigeria" was published in 2022. Journal: J Environ Public Health.

**Table 4:** Logistic regression analysis illustrating the influence of exposure to sex education and socio-demographic factors on having a sexual partner(s).

	*B*	S.E.	Wald	Sig.	Exp (B)
Place of residence					
Rural	RC				
Urban	0.20	0.87	1.31	0.25	2.71
Family type					
Extended	RC				
Nuclear	−0.60	0.54	1.23	0.27	0.55
Discussed sex issues with any or both parents					
No	RC				
Yes	1.37	0.58	5.56	0.02	3.93
Read things/discuss about sexual matter					
No	RC				
Yes	−1.04	1.06	0.97	0.33	0.35
Mother's occupation					
Civil servants	RC				
Farming/others	−2.15	0.84	6.50	0.01	0.12
Trading/services	−1.06	0.85	1.53	0.22	0.35
Father's occupation					
Civil servants	RC				
Farming/others	0.56	0.67	0.69	0.41	1.74
Trading/services	0.20	0.63	0.10	0.75	1.22
Age group					
15–19 years	RC				
≤14 years	−1.23	0.50	6.38	0.01	0.28
Gender					
Male	RC				
Female	0.09	0.53	0.03	0.87	1.09
Discussed sex issues with any relations					
No	RC				
Yes	−1.34	0.57	5.52	0.02	0.26
Frequency of reading/discussion matters					
Not at all	RC				
Very often	−1.32	0.54	5.98	0.01	0.27
Not often	−2.21	0.70	9.87	0.00	0.11
Rarely	−2.95	1.26	5.54	0.02	0.05
Constant	3.54	1.61	4.82	0.03	34.36
2 Log likelihood = 146.639; Overall percentage = 79.8	Nagelkerke R square = 0.463; Cox & Snell R square = 0.326				

Source: author's fieldwork (2021).

**Table 5:** Logistic regression analysis illustrating the influence of selected factors of exposure to sex education on having a sexual partner.

Selected variables	*B*	S.E.	Wald	Sig.	Exp(*B*)
Read things or discuss sexual matter					
No	RC				
Yes	−1.05	0.87	1.45	0.23	0.35
Discussed sex issues with any or both parents					
No	RC				
Yes	1.27	0.47	7.27	0.01	3.54
Discussed sex issues with any relations					
No	RC				
Yes	−1.27	0.45	8.06	0.01	0.28
Conceptual understanding of sex education					
Little	RC				
Good	−1.75	1.00	3.07	0.08	0.17
Average	−1.50	0.97	2.41	0.12	0.22
Frequency of discussion or reading					
Not at all	RC				
Very often	−1.01	0.45	5.01	0.03	0.36
Not often	−1.88	0.59	10.11	0.00	0.15
Rarely	−2.10	1.07	3.84	0.05	0.12
Source of first sex education					
Magazine/book	RC				
School	0.04	0.48	0.01	0.94	1.04
Family	1.81	1.64	1.21	0.27	6.09
Radio	−0.27	0.88	0.10	0.76	0.76
Television	−0.73	0.99	0.54	0.46	0.48
Social media	−1.99	1.19	2.79	0.10	0.14
Constant	1.85	1.0	3.43	0.06	6.35
Cox & Snell *R*^2^: 0.220	Nagelkerke *R*^2^: 0.311	2 log likelihood (177.35)		Overall percentage: 75.7	

Source: author's fieldwork (2021).

The article "Exposure to Sex Education and Its Effects on Adolescent Sexual Behavior in Nigeria" was published in 2022. Journal: J Environ Public Health.

## Data Availability

Data are available on request. Data for this study can be obtained directly from the Breast and Cervical Cancer Cluster of Covenant University. Contact details: Dr. Emmanuel O. Amoo, email: emma.amoo@covenantuniversity.edu.ng.
